# Roots of *Astragalus propinquus* Schischkin Regulate Transmembrane Iron Transport and Ferroptosis to Improve Cerebral Ischemia-Reperfusion Injury

**DOI:** 10.1155/2022/7410865

**Published:** 2022-08-02

**Authors:** Juan Chen, Donglai Ma, Jun Bao, Ying Zhang, Guoxing Deng

**Affiliations:** ^1^Graduate School, Hebei University of Chinese Medicine, Shijiazhuang 050200, Hebei, China; ^2^College of Pharmacy, Hebei University of Chinese Medicine, Shijiazhuang 050200, Hebei, China; ^3^Hebei Key Laboratory of Chinese Medicine Research on Cardio-Cerebrovascular Disease, Shijiazhuang 050200, China; ^4^College of Basic Medicine, Hebei University of Chinese Medicine, Shijiazhuang 050200, Hebei, China

## Abstract

**Background:**

The dried roots of the *Astragalus propinquus* Schischkin (RAP) plant, as a traditional Chinese medicine, has been widely used to treat stroke, cerebral ischemia, qi deficiency, and hypertension. Buyang Huanwu decoction is traditionally used to treat stroke in China for more than 200 years and has a significant effect on cerebral ischemia, and RAP is monarch medicine of Buyang Huanwu decoction. Therefore, this study was designed to observe the regulatory effect of RAP on transmembrane iron transporters and ferroptosis-related factors in cerebral ischemia-reperfusion injury (CIRI) in rats.

**Methods:**

Middle cerebral artery occlusion (MCAO) was used to block blood flow in the blood supply area of the middle cerebral artery in seventy male SD rats to induce focal CIRI to establish a rat model of CIRI. RAP was administered to explore the regulatory effect of RAP on iron transmembrane transport under the condition of CIRI. The infarct size was measured using 2,3,5-triphenyl-tetrazolium chloride (TTC) staining, the pathological structure of brain tissue was observed by HE staining, and neuronal injury was evaluated by Nissl staining after treatment. Then, changes in the iron transporters ferritin (Fn), ferritin heavy chain (FHC), ferritin light chain (FLC), transferrin (Tf), transferrin receptor (TfR), divalent metal transporter 1 (DMT1), L-type calcium channel (LTCC), transient receptor potential canonical 6 (TRPC6), and ferroportin 1 (FPN1) were observed by immunohistochemistry staining (IHC) and Western blotting. The expression of key factors of ferroptosis, including the membrane sodium-dependent cystine/glutamate antiporter System Xc^−^ (System Xc^−^) light chain subunit (XCT) and heavy chain subunit (SLC3A2), glutathione peroxidase 4 (GPX4), nuclear factor erythroid 2-related factor (NRF2), heme oxygenase-1 (HO-1), and iron-responsive element-binding protein 2 (IREB2) in the brain tissues of rats was assessed by Western blotting. RAP decreased the infarct size and neuronal injury after CIRI in rats. Similarly, RAP treatment regulated the expression of iron transporters. As such, RAP was able to reduce the expression of Fn, FHC, FLC, Tf, TfR, DMT1, and TRPC6 and increase the expression of FPN1 through a Tf/TfR-independent pathway after CIRI in rats.

**Conclusion:**

RAP stimulation inhibited ferroptosis by regulating the expression of the key ferroptosis factors XCT, SLC3A2, GPX4, NRF2, HO-1, and IREB2. In conclusion, RAP regulates transmembrane iron transport and ferroptosis to improve CIRI.

## 1. Introduction

Ischemic stroke is a destructive brain injury and one of the leading causes of death and physical disability worldwide [1, 2]. Reperfusion is an effective treatment for cerebral ischemia. However, the damage to ischemic brain tissue is further aggravated when the blood restores perfusion, and this process is defined as CIRI. Oxidative stress is involved in the entire pathological process, and iron plays a key role in CIRI.

Iron overload occurs resulting in DNA damage, lipid peroxidation, neuronal apoptosis, and mitochondrial autophagy in CIRI [3]. Under normal conditions, iron enters cells mainly through a Tf/TfR-dependent pathway. Cells acquire iron from Tf [4], which binds iron with a high affinity to form a unique chelated form of iron. Transferrin receptors (TfRs) are involved in the uptake of Tf-bound iron from the plasma into cerebral endothelial cells; among these receptors, TfR1 is essential for cellular iron uptake and is widely distributed in neurons [5, 6]. Fn is the main iron storage protein, which is composed of two subunit types, the H- and L-chains [7]. Under iron overload conditions, Tf/TfR-independent pathways become the major pathways by which iron enters cells due to the oversaturation of the Tf/TfR-dependent pathway [4, 8, 9]. Tf/TfR-independent iron transmembrane transporters mainly include: DMT1, LTCC, TRPC6, FPN1 [10–12].

Ferroptosis plays an important role in the occurrence and development of ischemic stroke by affecting iron metabolism and lipid peroxidation [13, 14]. The loss of GPX4 activity is the main cause of ferroptosis. The activity of GPX4 is controlled by glutathione (GSH), and the availability of cysteine is essential for the synthesis of GSH. Cells import cystine using System Xc^−^, which consists of XCT and SLC3A2 and is mainly responsible for intracellular cystine uptake [15, 16]. There is increasing evidence that SLC3A2 is also important in preventing excessive lipid peroxidation in cells [16, 17]. Recent studies have shown that IREB2 and HO-1 also play important roles in ferroptosis [18, 19].

Thrombolytic and neuroprotective therapies are recommended for patients suffering from ischemic stroke. Thrombolytic therapy is one of the most effective treatment measures, but it has strict time window restrictions and side effects. Neuroprotective agents are considered to be the most promising drugs, and the purpose of their treatment is to reduce brain tissue injury and inhibit nerve cell death after cerebral ischemia reperfusion. Edaravone is an antioxidant free radical scavenger, but it has a single therapeutic target and also causes various adverse reactions [20].

The dried roots of plant *Astragalus propinquus* Schischkin (RAP) is a traditional Chinese medicine (TCM), also known as Huang Qi or *Radix Astragali* [21, 22]. Its plant name has been checked with https://www.theplantlist.org. RAP was first recorded in the earliest Chinese pharmacy monograph “Shen Nong's Herbs” with more than 2000 years history [21]. According to Chinese medicine theory, RAP is capable of raising yang qi and tonifying the spleen and lung qi, thereby facilitating urination and reducing edema [23]. In TCM, RAP has been widely used to treat stroke, cerebral ischemia, qi deficiency, hypertension, and many other diseases [24–27]. Buyang Huanwu decoction (BHD), a classic TCM formula, was first created by Qingren Wang in the book Correction of Errors in Medical Classics (Yi Lin Gai Cuo) [28]. It has the effect of tonifying qi, promoting blood circulation, and opening the meridians and collaterals. It has been traditionally used to treat stroke in China for 200 years and has a significant effect on cerebral ischemia [29, 30]. BHD consists of seven herbs: *Astragalus propinquus* Schischkin (Huangqi) 120 g, *Angelica sinensis* (Oliv.) Diels (Danggui) 6 g, *Paeonia lactiflora* Pall (Chishao) 4.5 g, *Ligusticum striatum* DC. (Chuanxiong) 3 g, *Lumbricus* (Dilong) 3 g, *Prunus persica* (L.) Batsch (Taoren) 3 g, and *Carthamus tinctorius* L. (Honghua) 3 g, among which RAP is monarch medicine, with a dosage of up to 120 g [30–33]. In this study, we adopted the same dose of RAP in BHD.

Modern pharmacological studies show that RAP possesses a variety of chemical components, mainly including *Astragalus* polysaccharides, saponins, flavonoids, and amino acids. The 2020 edition of “Chinese Pharmacopoeia” takes the content of calycosin and astragaloside as the quality control standard for RAP [34]. Currently, the commercially available dosage forms of RAP in China mainly include two types, granule and injection. RAP granule is included in the “Standards Issued by the Ministry of Traditional Chinese Medicine” with standard number of WS3-B-2224-96, and is a full-component extract of A*stragalus propinquus* Schischkin dried roots [35]. RAP injection is a sterilized aqueous solution prepared by extracting the dried roots of *Astragalus propinquus* Schischkin. Compared with granule, it has the characteristics of high absorption and availability and rapid curative effect [36].

Experimental studies confirm that RAP and Astragaloside IV can alleviate brain tissues in ischemia-reperfusion injured rats [37]. *Astragalus* polysaccharide upregulates hepcidin and reduces iron overload in mice [38]. Moreover, *Astragalus* polysaccharide treatment significantly reduces apoptosis, regulates oxidative stress, and upregulates GSH peroxidase activity [39]. Calycosin is an effective monomer of RAP and can protect brain nerve cells from CIRI through antioxidant, antiapoptotic, anti-inflammatory, and autophagic activities [40, 41]. Therefore, we hypothesized that RAP has a neuroprotective effect on CIRI, which may be related to its regulation of transmembrane iron transport and improvement of ferroptosis in the brain.

In the present study, we first determined the neuroprotective effect of RAP in CIRI model rats. Then, we clarified the mechanism of RAP in CIRI iron injury and identified the molecular targets of RAP and its monomer calycosin in transmembrane iron transport and ferroptosis. In addition, we compared the difference in the efficacy of granule and injection of RAP.

## 2. Materials and Methods

### 2.1. Ethics and Animals

All experimental procedures were approved by the Ethics Committee of Hebei University of Chinese Medicine (Shijiazhuang, China). In this study, 70 SD healthy male rats weighing 120–150 g were purchased from Beijing Vital River Laboratory Animal Technology Co., Ltd. (license number: SCXK, Beijing, 2016-0006, ethics number: DWLL2020080). All rats were housed with free access to food and water at a constant temperature of 22 ± 2°C under a 12 h light/dark cycle with a relative humidity of 40–60%. All animals were treated as humanely as possible to alleviate the pain suffered during the experiment.

### 2.2. Establishment of an MCAO and Reperfusion Model in Rats

The MCAO model was established according to methods outlined by Longa [42]. The rats were anesthetized with 1% pentobarbital sodium (50 mg/kg), and then the right common carotid artery (CCA), external carotid artery (ECA), and internal carotid artery (ICA) were bluntly separated. The ECA was ligated, and then the proximal end of the CCA and the ICA were clamped with arterial clamps. A 45° incision was made in the ECA, and a round 4-0 single wire bolt was gently inserted at the end of the head into the ICA until slight resistance was encountered (18 mm). After 2 hours of ischemia, the thread was gently pulled out to restore cerebral blood circulation. In the sham group, only the skin was cut open, and the right CCA was bluntly separated, after which the incision was sutured without the ischemia-reperfusion procedure.

### 2.3. Groups and Drug Administration

All rats were randomly divided into 7 groups: the sham group, model group, RAP granule group, RAP injection group, calycosin group, edaravone group, and deferoxamine group. The CIRI model was established in all groups except for the sham group. The sham group and model group received a single intraperitoneal injection of 0.9% NaCl; the RAP granule group received a stomach feeding of 2.5 g/kg/d RAP granule (SHINEWAY Pharmaceutical Group Co., Ltd., Shijiazhuang, China, 20071141); the RAP injection (SHINEWAY Pharmaceutical Group Co., Ltd., Shijiazhuang, China, 200827C1) group, calycosin (purity >98.00%, GlpBio Technology Inc, Montclair, CA, USA, 20575-57-9) group, edaravone (Jilin Province Boldere Pharmaceutical Co., Ltd., Jilin, China, 01–2000031) group and deferoxamine (purity >98.00%, GlpBio Technology Inc, Montclair, CA, USA, 54078-29-4) group were intraperitoneally injected with RAP (2 mL/kg/d), calycosin (10 mg/kg/d), edaravone (6.3 mg/kg/d), and deferoxamine (70 mg/kg/d), respectively. These administrations were given 7 days prior to the operation and 3 days following reperfusion, as shown in Figure 1.

### 2.4. High performance Liquid Chromatography (HPLC) Analysis

The RAP granule/RAP injection was evaluated by high performance liquid chromatography (HPLC) analysis. Briefly, HPLC-ELSD was performed using Agilent-1260 (Agilent, California, USA) equipped with Thermo BDS Hypersil C-18 (250 mm × 4.6 mm, 5 *μ*m). The column temperature was 30°C, the nebulizer temperature was 40°C, the nitrogen flow rate was 1.6 mL/min, and the injection volume was 10 *μ*L. The mobile phase was eluted with acetonitrile (A) and 0.2% acetic acid solution (B) in the gradient mode. The proportion of acetonitrile varied from 20% to 40% within 30 min (0–20 min, 20%–40% A; 20–30 min, 40% A) at a flow rate of 0.9 mL/min.

### 2.5. Staining and Measurement of Brain Infarct Size

The brain was cut coronally into five 2 mm-thick sections and immersed in TTC for 20 min at 37°C in the dark. Then, the brain slices were removed, the TTC staining solution was discarded, and PBS was added to stop the staining. After removing the brain slices, they were placed in a tissue fixing solution, and photos were taken after fixing for 24 hours. After the imaging was completed, Image-ProPlus 6.0 analysis software (Media Cybemetics, U.S.A.) was used to measure the pixel area of each tissue in each picture and the corresponding infarcted pixel area, using pixels as the standard unit. Then, the proportion of tissue infarcted area (%) was calculated with the following equation:

(1) $$\begin{array}{c} \text{Infarct size}\left(\%\right)=\frac{\text{infarcted pixel area}}{\text{tissue pixel area}}\times 100. \end{array}$$

### 2.6. HE Staining

Paraffin slices were dewaxed in water and then xylene twice, 5 min each time, rehydrated in an alcohol gradient of 100%, 95%, and 80%, 5 min each time, and then washed with tap water. The slices were immersed in hematoxylin for 3 minutes, followed by washing with tap water 2-3 times, and then in hydrochloric acid alcohol differentiation solution, followed by washing with tap water. The slices were incubated in blue solution for 5–15 s, followed by washing with tap water, and then stained with eosin for 10 s, followed by washing with tap water. The slices were then incubated in 80% alcohol for 5 min, 90% alcohol for 5 min, 100% alcohol for 5 min, and then xylene. The slices were sealed with neutral gum, after which they were observed by optical microscopy, and the images were collected.

### 2.7. Nissl Staining

The sections were immersed in xylene two times for 15 min each, placed into a series of ethanol concentrations starting from 50% to 100% for 5 min each and then rinsed with distilled water 3 times. Subsequently, the sections underwent Nissl staining according to standard protocols. Then, the pathological changes in the brain tissue were observed under a microscope.

### 2.8. IHC  and  Western Blotting

In the present study, IHC and Western blotting were carried out as described in our previous study [43, 44]. For IHC, the paraffin-embedded sections were dewaxed in xylene, rehydrated in a graded alcohol series (100%, 95%, and 80%), and then washed 3 times with distilled water. Subsequently, the sections were blocked with 3% H_2_O_2_ at 37°C for 10 min and washed 5 times with PBS. Then, the sections were heated in a microwave oven in sodium citrate buffer for 20 min for antigen retrieval and washed 5 times with PBS. Then, the slices were incubated with primary antibodies overnight at 4°C, using the following primary antibodies: anti-Fn (1 : 1000; WG3336219F); anti-Tf (1 : 1000; CC02161); anti-TfR (1 : 1000; 33r7946); anti-DMT1 (1 : 1000; 89p5609); anti-LTCC (1 : 1000; 59v9215); anti-TRPC6 (1 : 1000; AD112056); and anti-FPN1 (1 : 1000; 89a3321). The next day, the sections were incubated with a secondary antibody at 37°C for 1 hour, DAB for development of color, and hematoxylin for counterstaining after washing with running water, and then washed back to blue with running water. Finally, the stained sections were observed under a light microscope.

For Western blotting, the brain tissues were homogenized by using RIPA lysis buffer to extract total protein. The proteins were separated by SDS-PAGE and then transferred from the gel to nitrocellulose membranes. The membranes were blocked with 5% skim milk and then incubated overnight at 4°C with the following primary antibodies: anti-FHC (1 : 1000; 32j4044); anti-FLC (1 : 1000; 89P1630); anti-Tf (1 : 1000; CC02161); anti-TfR (1 : 1000; 33r7946); anti-DMT1 (1 : 1000; 89p5609); anti-TRPC6 (1 : 1000; AD112056); and anti-FPN1 (1 : 1000; 89a3321). The membranes were then washed 3 times with TBST and incubated with the secondary antibody for 1 hour. Protein band densities were scanned and analyzed by using a computerized image analysis system and ImageJ.

### 2.9. Ferroptosis Index Assessment by Western Blot

The brain tissues were homogenized by using RIPA lysis buffer to extract total protein. The proteins were separated by SDS-PAGE and then transferred from the gel to nitrocellulose membranes. The membranes were blocked with 5% skimmed milk and then incubated overnight at 4°C with the following primary antibodies: anti-XCT (1 : 5000; GR3337924-9); anti-SLC3A2 (1 : 1000; 14e3479); anti-GPX4 (1 : 1000; 78p5366); anti-NRF2 (1 : 1000; 65m9929); anti-IREB2 (1 : 1000; WG3335638A), and anti-HO-1 (1 : 1000; BJ02265489). The membranes were then washed 3 times with TBST and incubated with the secondary antibody for 1 hour. Protein band densities were scanned and analyzed by using a computerized image analysis system and ImageJ.

### 2.10. Statistical Analysis

Statistical analysis of the data was performed using SPSS (IBM SPSS Statistics v 26.0.0). All data satisfying normality are expressed as the mean ± SEM. The differences among the multiple groups were evaluated by one-way ANOVA, followed by LSD for comparison of two groups. The results were considered statistically significant at *P* < 0.05 and at *P* < 0.01.

## 3. Results

### 3.1. HPLC Analysis of RAP Granule and RAP Injection

The RAP granule and RAP injection were evaluated by high performance liquid chromatography (HPLC) analysis to identify the presence of Calycosin-7-O-glucoside and Astragaloside A according to their retention times (Figures 2(a) and 2(b)).

### 3.2. RAP Attenuates Ischemic Injury after MCAO

To explore the effect of RAP on CIRI, the cerebral infarction area in rats after MCAO and after administration of various agents was observed. As shown in Figures 3(a) and 3(b) and Table 1, compared with the sham group, the cerebral infarction area in the model group increased significantly (*P* < 0.01). Compared with the model group, the area of cerebral infarction in the RAP granule group, RAP injection group, and edaravone group decreased, especially in the RAP granule group (*P* < 0.01). These results show that RAP can alleviate the brain injury caused by ischemia.

### 3.3. Results of HE Staining of the Hippocampal CA3 Region

Under a pathological microscope, the hippocampal CA3 region of rats in the sham group was characterized by an intact cellular structure and orderly tissue arrangement. In the model group, the arrangement of the brain tissue was disordered, the structure of the neurons was seriously damaged, and some nerve cells were necrotic. The RAP granule group, RAP injection group and calycosin group showed effective reductions in neuronal injury, and the tissue arrangement in these groups was significantly better than that in the model group (Figure 4(a)).

### 3.4. Neuronal Apoptosis in the Hippocampal CA3 Region

According to the results of the Nissl staining, the hippocampal CA3 region of the rats in the sham group was characterized by an intact cell structure, regular nuclear morphology, clear nucleoli, and abundant Nissl bodies in the cytoplasm (*P* < 0.01). However, after MCAO, the arrangement of cells in the CA3 region of the hippocampus was loose, the cell bodies of some residual neurons shrank, the nuclei were pyknotic, and the Nissl bodies in the cytoplasm were decreased. After drug treatment, the neuronal injury was improved, the number of Nissl bodies in the cytoplasm was increased, and the differences were most significant in the RAP granule group and the RAP injection group (*P* < 0.05, Figure 4(b), Table 2).

### 3.5. Expression of Iron Transporters in the Different Treatment Groups

To verify the regulatory effect of RAP on transmembrane iron transport, IHC and Western blotting were used to observe the changes in iron transporters (storage proteins Fn, FHC, and FLC, transfer proteins Tf, TfR, DMT1, TRPC6, and LTCC, and efflux protein FPN1) before and after administration of the various agents.

#### 3.5.1. IHC and Western Blot Results

*(1) Effect of RAP on Fn, FHC, and FLC Protein Expression.* According to the results of the IHC, the expression level of Fn protein in the model group was significantly higher than that in the sham group (*P* < 0.01). Compared with the model group, the expression of Fn protein decreased in the RAP granule group, RAP injection group, and calycosin group, especially in the RAP granule group (*P* < 0.01, Figures 5(a) and 5(b), Table 3). Western blot results in Figure 5(c) and Table 3 show that compared with the sham group, the expression level of FHC protein in the model group was significantly higher (*P* < 0.01). Compared with the model group, the expression level of FHC protein in the RAP granule group, RAP injection group, and calycosin group decreased, especially in the RAP injection group (*P* < 0.01). As shown in Figure 5(d) and Table 3, compared with the sham group, the expression level of FLC protein in the model group was significantly higher (*P* < 0.01). Compared with the model group, the expression level of FLC protein in the RAP granule group, RAP injection group, and calycosin group decreased, especially in the RAP granule group (*P* < 0.01).

*(2) Effect of RAP on LTCC Protein Expression.* As shown in Figures 6(a1) and 6(a2) and Table 4, compared with the sham group, the expression level of LTCC protein in the model group increased (*P* < 0.01), and compared with the model group, the expression level of LTCC protein in the RAP granule group, RAP injection group, and calycosin group decreased, especially in the RAP injection group (*P* < 0.05).

*(3) Effect of RAP on Tf Protein Expression.* Compared with the sham group, the expression level of Tf protein in the model group increased (*P* < 0.01), and compared with the model group, the expression level of Tf protein in the RAP granule group, RAP injection group, and calycosin group decreased, especially in the RAP granule group (*P* < 0.01, Figure 6(b1), Table 5). Western blot results showed that the expression level of Tf protein in the model group (0.894 ± 0.04) was significantly higher than that in the sham group (0.561 ± 0.05) (*P* < 0.01). Compared with the model group, the expression level of Tf protein in the RAP granule group (0.565 ± 0.08), RAP injection group (0.554 ± 0.07), and calycosin group (0.673 ± 0.06) decreased, especially in the RAP injection group (*P* < 0.01, Figure 6(b2)).

*(4) Effect of RAP on TfR Protein Expression.* As shown in Figure 6(c1) and Table 5, compared with the sham group (*P* < 0.01), the TfR protein expression level in the model group was increased. Compared with the model group, the TfR protein expression level of the RAP granule group, RAP injection group, and calycosin group decreased, with the RAP granule group decrease being the most significant (*P* < 0.01). Western blot results showed that the expression level of TfR protein in the model group (0.838 ± 0.08) was significantly higher than that in the sham group (0.569 ± 0.05) (*P* < 0.01). Compared with the model group, the expression level of TfR protein in the RAP granule group (0.450 ± 0.06), RAP injection group (0.469 ± 0.06), and calycosin group (0.558 ± 0.08) decreased, especially in the RAP granule group (*P* < 0.01, Figure 6(c2)).

*(5) Effect of RAP on DMT1 Protein Expression*. As shown in Figure 6(d1) and Table 5, compared with the sham group, the DMT1 protein expression level in the model group was increased (*P* < 0.01). Compared with the model group, the protein expression level of DMT1 in the RAP granule group, RAP injection group, and calycosin group was decreased, and the difference was statistically significant in the RAP injection group (*P* < 0.01). Western blot results showed that compared with the sham group (0.612 ± 0.07), the expression level of DMT1 protein in the model group (0.809 ± 0.05) increased (*P* < 0.05). Compared with the model group, the expression level of DMT1 protein in the RAP granule group (0.594 ± 0.05), RAP injection group (0.635 ± 0.06), and calycosin group (0.633 ± 0.05) decreased, especially in the RAP granule group (*P* < 0.05, Figure 6(d2)).

*(6) Effect of RAP on TRPC6 Protein Expression.* As shown in Figure 6(e1) and Table 5, compared with the sham group, the expression level of TRPC6 protein in the model group increased (*P* < 0.01), and compared with the model group, the expression level of TRPC6 protein in the RAP granule group, RAP injection group, and calycosin group decreased, especially in the RAP granule group (*P* < 0.01). Western blot results showed that compared with the sham group (0.580 ± 0.08), the expression level of TRPC6 protein in the model group (0.867 ± 0.08) increased (*P* < 0.05). Compared with the model group, the expression level of TRPC6 protein in the RAP granule group (0.494 ± 0.06), RAP injection group (0.555 ± 0.04), and calycosin group (0.577 ± 0.06) decreased, especially in the RAP granule group (*P* < 0.01, Figure 6(e2)).

*(7) Effect of RAP on FPN1 Protein Expression.* As shown in Figure 6(f1) and Table 5, compared with the sham group, the expression level of FPN1 protein in the model group decreased (*P* < 0.01), and compared with the model group, the expression level of FPN1 protein in the RAP granule group, RAP injection group, and calycosin group increased, especially in the RAP granule group (*P* < 0.05). Western blot results showed that compared with the sham group (0.750 ± 0.07), the expression level of FPN1 protein in the model group (0.447 ± 0.08) decreased (*P* < 0.05). Compared with the model group, the expression level of FPN1 protein in the RAP granule group (0.779 ± 0.08), RAP injection group (0.784 ± 0.11), and calycosin group (0.924 ± 0.12) increased, especially in the calycosin group (*P* < 0.01, Figure 6(f2)).

#### 3.5.2. The Main Factors of the Ferroptosis Signaling Pathway Include XCT, SLC3a2, IREB2, NRF2, HO-1, and GPX4

GPX4 plays an important role in ferroptosis [45]

*(1) Effect of RAP on Expression of the XCT Protein*. As shown in Figure 7(a), compared with the sham group (0.835 ± 0.04), the expression level of XCT protein in the model group (0.529 ± 0.10) decreased (*P* < 0.01), and compared with the model group, the expression level of XCT protein in the RAP granule group (0.767 ± 0.07), RAP injection group (0.853 ± 0.03), and calycosin group (0.857 ± 0.04) increased, especially in the calycosin group (*P* < 0.01).

*(2) Effect of RAP on Expression of the SLC3A2 Protein.* As shown in Figure 7(b), compared with the sham group (0.766 ± 0.06), the expression level of SLC3A2 protein in the model group (0.456 ± 0.06) decreased (*P* < 0.01), and compared with the model group, the expression level of SLC3A2 protein in the RAP granule group (0.773 ± 0.07), RAP injection group (0.847 ± 0.04), and calycosin group (0.883 ± 0.09) increased, especially in the calycosin group (*P* < 0.01).

*(3) Effect of RAP on Expression of the GPX4 Protein.* As shown in Figure 7(c), compared with the sham group (0.694 ± 0.05), the expression level of GPX4 protein in the model group (0.466 ± 0.04) decreased (*P* < 0.05), and compared with the model group, the expression level of GPX4 protein in the RAP granule group (0.719 ± 0.06), RAP injection group (0.667 ± 0.06), and calycosin group (0.784 ± 0.05) increased, especially in the calycosin group (*P* < 0.01).

*(4) Effect of RAP on Expression of the NRF2 Protein.* As shown in Figure 7(d), compared with the sham group (0.605 ± 0.06), the expression level of NRF2 protein in the model group (0.350 ± 0.07) decreased (*P* < 0.05), and compared with the model group, the expression level of NRF2 protein in the RAP granule group (0.686 ± 0.04), RAP injection group (0.702 ± 0.11), and calycosin group (0.653 ± 0.09) increased, especially in the RAP injection group (*P* < 0.01).

*(5) Effect of RAP on Expression of the HO-1 Protein.* As shown in Figure 7(e), compared with the sham group (0.622 ± 0.03), the expression level of HO-1 protein in the model group (0.387 ± 0.08) decreased (*P* < 0.05), and compared with the model group, the expression level of HO-1 protein in the RAP granule group (0.587 ± 0.07), RAP injection group (0.543 ± 0.06), and calycosin group (0.696 ± 0.06) increased, especially in the calycosin group (*P* < 0.01).

*(6) Effect of RAP on Expression of the IREB2 Protein.* As shown in Figure 7(f), compared with the sham group (0.469 ± 0.05), the IREB2 protein expression level was increased in the model group (0.781 ± 0.04) (*P* < 0.01). Compared with the model group, the protein expression level of IREB2 in the RAP granule group (0.554 ± 0.08), RAP injection group (0.619 ± 0.08), and calycosin group (0.537 ± 0.07) decreased, especially in the calycosin group (*P* < 0.05).

## 4. Discussion

Ischemic brain tissue injury is further aggravated after the restoration of blood perfusion, otherwise known as CIRI, and its pathophysiological process is a cascade reaction of multiple linked factors and pathways. The recovery of neural function is helpful for alleviating CIRI [46]. Previous studies have found that RAP contains a variety of active components acting on the cardiovascular system and cerebral vasculature, which can effectively restore nerve function damage [37, 41, 47]. In this study, it was found that after 2 hours of cerebral ischemia and reperfusion, the rats showed obvious neurological damage: the size of cerebral infarction on the ischemic side increased, the arrangement of brain tissue was disordered, the structure of the neurons was seriously damaged, and some cells were necrotic. However, RAP treatment significantly reduced the incidence of cerebral infarction on the ischemic side of rats after MCAO, the arrangement of brain tissue was significantly better than that of the CIRI group, and the neuronal damage was effectively reduced, consistent with previous studies [37, 48, 49].

Traditional Chinese medicine, with its ability to affect multiple targets and pathways, has prominent advantages in the prevention and treatment of CIRI. RAP is a commonly used Chinese herbal medicine for the treatment of cardio-cerebrovascular diseases. Modern pharmacological studies have shown that RAP contains a variety of active ingredients, such as *Astragalus* polysaccharides, astragalosides, and *Astragalus* flavonoids, which have antioxidant, anti-inflammatory, and antiapoptotic effects and can treat ischemic cardio-cerebrovascular diseases. Two dosage forms, RAP granules and RAP injection, are widely used to treat ischemic cerebrovascular diseases in the clinic [50, 51]. As an effective component of RAP, calycosin has a neuroprotective effect on CIRI in rats, protects the inherent antioxidant function of cells, prevents excitotoxicity of nerve cells caused by Glu, and has a strong ability to scavenge free radicals [52–54]. In addition, our previous studies have shown that astragaloside IV has a protective effect in liver injury caused by iron overload [55].

Brain iron homeostasis is critical to the normal physiological function of neurons. CIRI can lead to iron deposition in neurons, which catalyzes the production of a large number of free radicals, leads to a series of brain injuries (such as oxidative damage, edema, and aggravation of infarction), and finally induces cell death [56–58]. Studies have shown that iron overload aggravates CIRI injury [59] and that the hippocampus is the region most sensitive to CIRI [60]. Fn is responsible for storing excess iron in cells to avoid the production of free radicals from free iron. Studies have shown that the expression of the iron storage proteins H-ferritin and L-ferritin increased significantly in the hippocampus on the ischemic side of the brain [60, 61]. In this study, we found that expression of the storage protein Fn (FHC and FLC) increased significantly in the hippocampal CA3 region of rats after 2 hours of ischemia and reperfusion, and the expression levels of Fn, FHC, and FLC decreased significantly after treatment with RAP, which was consistent with a previous study. It is suggested that RAP can reduce the content of the iron storage protein Fn (FHC and FLC) in the brain and relieve brain injury after CIRI.

In the iron transmembrane transport system, the Tf/TfR-dependent pathway plays an important role and is closely related to maintaining iron homeostasis in the brain. Tf is the main iron transporter and requires receptor-mediated endocytosis to cross the blood–brain barrier [62–64]. TfR exists in cerebral vascular endothelial cells and binds transferrin-bound iron [63, 64]. Previous studies found that the expression of TfR increased after CIRI [65], and MCAO stimulation increased the expression of TfR in the brain, resulting in abnormal expression of iron-related proteins and inhibiting the changes after administration [66]. In this study, we observed that the expression of Tf and TfR increased after 2 hours of cerebral ischemia and reperfusion, while the expression of Tf and TfR decreased after treatment with RAP, which was consistent with a previous study. The results showed that RAP can reduce iron import in the brain by inhibiting the high expression of Tf and TfR, promote the balance of brain iron, and prevent the occurrence of brain iron overload after CIRI.

In addition, iron transport across cell membranes may involve in Tf/TfR-independent pathways, such as DMT1, LTCC, TRPC6, and FPN1. In the transferrin cycle, Tf binds to TfR1 on the cell surface, followed by endocytosis and acidification, resulting in iron release from transferrin. The free Fe^3+^ is reduced to Fe^2+^ in the endosome and transported to the cytoplasm through DMT1. In the iron overloaded state, supersaturation of transferrin exists in the form of nontransferrin bound iron (NTBI), and the uptake of NTBI needs to be mediated by NTBI transporters such as DMT1, LTCC, and TRPC6 [67]. Excessive intake of NTBI and lack of effective excretion can lead to the production of reactive oxygen free radicals [68]. In a study on nifedipine, an LTCC blocker, it was found to stimulate DMT1-mediated iron transport and reduce iron overload, indicating that LTCC blockers could regulate DMT1-mediated iron transport [69]. Iron toxicity induced by brain iron overload can increase the infarct size in MCAO rats [70]. The imbalance between iron input proteins DMT1, LTCC, TRPC6, and output protein FPN1 is considered to be the main trigger of brain iron disorder after cerebral ischemia [57, 68, 71, 72]. In this study, the expression of DMT1, LTCC, and TRPC6 increased after 2 hours of cerebral ischemia reperfusion in rats. After treatment with RAP and deferoxamine, the expression of DMT1, LTCC, and TRPC6 decreased. Deferoxamine can reduce the size of cerebral infarction and decrease the level of brain iron after MCAO in rats. RAP has an iron removal effect similar to that of deferoxamine, suggesting that RAP can effectively reduce iron deposition in neurons and can alleviate CIRI by alleviating iron toxicity caused by brain iron deposition after cerebral ischemia, which is consistent with previous studies.

Moreover, one transporter, FPN1, capable of transferring iron out of cells, has been found in the brain thus far [11, 12]. In this study, the expression of FPN1 in the hippocampal CA3 region of rats stimulated by MCAO decreased, and the expression of FPN1 increased after treatment with RAP and deferoxamine. It has been reported that the increase in brain iron after CIRI is related to the abnormal iron output mediated by FPN [13]. Tau knockout can protect young mice from MCAO-induced brain iron deposition and reduce CIRI. With increasing age, drugs to promote iron efflux should be used to reduce CIRI. This effect is consistent with the results of this study, suggesting that RAP has a similar effect as deferoxamine by upregulating the expression of FPN1, increasing brain iron efflux, promoting brain iron metabolism balance, and ultimately reducing CIRI.

Ferroptosis is a new type of iron-dependent programmed cell death that is characterized by iron-dependent lipid peroxidation [73]. Recent studies have found that ferroptosis plays an important role in the occurrence and development of ischemic stroke by affecting iron metabolism or lipid peroxidation. System Xc^−^, composed of XCT and SLC3A2, is critical in ferroptosis [17, 74–76]. Studies have shown that inhibition of XCT and SLC3A2 expression can promote tumor cell lipid peroxidation and ferroptosis [76, 77]. In this study, MCAO was shown to stimulate a reduction in XCT and SLC3A2 protein expression levels in rats. After treatment, RAP showed a similar effect to deferoxamine and increased the protein expression of XCT, SLC3A2, and GPX4. This result is consistent with previous studies.

In addition, iron metabolism is required for the accumulation of lipid peroxides and the execution of ferroptosis [78]. One study found that the ferroptosis inhibitor ferrostatin-1 could reduce iron and ROS accumulation and downregulate the ferroptosis-related gene IREB2 to further inhibit ferroptosis [79]. In this study, it was found that compared with the sham group, the expression of IREB2 protein in MCAO rats increased and that the expression of IREB2 protein decreased after treatment with RAP and deferoxamine. This further indicates that RAP may activate System Xc^−^ (XCT, SLC3A2), enhance the activity of GPX4, inhibit lipid peroxidation, downregulate the expression of IREB2, regulate iron metabolism, and inhibit the occurrence of ferroptosis. Previous studies have shown that the NRF2/HO-1 pathway plays an important role in CIRI and ferroptosis [80, 81]. NRF2 is a gene related to ferroptosis that plays an antioxidant role and inhibition of ferroptosis by activating downstream antioxidant genes, such as HO-1 and GPX4 [78, 82, 83]. HO-1 is a downstream signaling molecule that regulates the expression of NRF2 after entering the nucleus [84]. GPX4 is a gene mediated by the NRF2 transcription pathway [85]. In this study, we found that the protein expression of NRF2, HO-1, and GPX4 decreased after MCAO stimulation. After treatment with RAP and deferoxamine, the protein expression of NRF2, HO-1, and GPX4 increased. It is suggested that RAP has an effect of iron removal similar to deferoxamine, which can prevent ferroptosis after CIRI by regulating ferroptosis-related proteins. This result is consistent with previous studies [80]. Based on the above research results, we found that RAP granule was more effective than RAP injection on iron transmembrane transporters, while calycosin has an obvious effect on ferroptosis.

## 5. Conclusions

Generally, brain iron transmembrane transporters are involved in the process of CIRI. RAP downregulated Tf, TfR, Fn, FHC, FLC, DMT1, LTCC, and TRPC6, upregulated FPN1, regulated the expression of iron transporters, and played a role in the prevention and treatment of CIRI. We also found that the key factors of ferroptosis were involved in ischemic stroke. Calycosin inhibited the occurrence of ferroptosis by regulating the expression of XCT, SLC3A2, GPX4, NRF2, HO-1, and IREB2.

## Figures and Tables

**Figure 1:** Diagram of the procedures using medication for treatment of CIRI.

**Figure 2:** The main active constituents of RAP granule and RAP injection. (a) RAP granule; (b) RAP injection.

**Figure 3:** Effect of RAP on cerebral infarct size in rats after CIRI induced by MCAO determined by TTC staining. (a) One representative image of each of the seven groups is shown; (b) Statistical results of cerebral infarct size in the seven groups (n = 5). ^*∗∗*^*P* < 0.01 vs. sham group, ^#^*P* < 0.05, ^##^*P* < 0.01 vs. model group.

**Figure 4:** (a) Representative images of HE staining of the hippocampal CA3 area of the ischemic side in the rats (×400). (b) Representative images of Nissl staining in the hippocampal CA3 region (×400). Black arrow: necrotic neuron. Scale bar = 100 *μ*m. Statistical results of the Nissl staining in the seven groups (*n* = 5). ^*∗∗*^*P* < 0.01 vs. sham group, ^#^*P* < 0.05 vs. model group.

**Figure 5:** Effect of RAP on the expression of Fn, FHC, and FLC after CIRI. (a) One representative image of each of the seven groups is shown (IHC, ×400). (b) Statistical results of Fn protein expression in the seven groups (*n* = 5). (c) Statistical results of FHC protein expression in the seven groups (*n* = 5). (d) Statistical results of FLC protein expression in the seven groups (*n* = 5). Scale bar = 100 *μ*m. ^*∗∗*^*P* < 0.01 vs. sham group; ^#^*P* < 0.05 and ^##^*P* < 0.01 vs. model group.

**Figure 6:** Effect of RAP on the expression of LTCC, Tf, TfR, DMT1, TRPC6, and FPN1 after CIRI. Representative IHC images (a1, b1, c1, d1, e1, f1) (×400). Scale bar = 100 *μ*m. Statistical results of the seven groups (a2, b2, c2, d2, e2, f2) (*n* = 5; ^*∗*^*P* < 0.05, ^*∗∗*^*P* < 0.01 vs. sham group; ^#^*P* < 0.05 and ^##^*P* < 0.01 vs. model group).

**Figure 7:** Effect of RAP on the expression of XCT, SLC3A2, GPX4, NRF2, HO-1, and IREB2 after CIRI. Statistical results of the WB experiments in the seven groups. Data are expressed as the mean ± SEM, *n* = 5. ^*∗*^*P* < 0.05, ^*∗∗*^*P* < 0.01 vs. sham group; ^#^*P* < 0.05, ^##^*P* < 0.01 vs. model group.

**Table 1:** Effect on cerebral infarct size in rats after CIRI induced by MCAO determined by TTC staining.

Group	Dose (g·kg^−1^)	Infarct size (%)
Sham		15.42 ± 4.90
Model		44.64 ± 7.73^*∗∗*^
RAP granule	2.5 g/kg	18.63 ± 5.41^##^
RAP injection	2 ml/kg	22.00 ± 6.76^#^
Calycosin	10 mg/kg	29.55 ± 6.99
Edaravone	6.3 mg/kg	23.96 ± 5.39^#^
Deferoxamine	70 mg/kg	30.37 ± 7.06

Data are expressed as the mean ± SEM, *n* = 5. ^*∗∗*^*P* < 0.01 vs. sham group. ^#^*P* < 0.05 and ^##^*P* < 0.01 vs. model group.

**Table 2:** Comparison of Nissl body counts in each group.

Group	Dose (g·kg^−1^)	Nissl body counts
Sham		8.40 ± 1.78
Model		3.20 ± 1.02^*∗∗*^
RAP granule	2.5 g/kg	7.40 ± 0.98^#^
RAP injection	2 ml/kg	7.40 ± 1.40^#^
Calycosin	10 mg/kg	6.00 ± 0.84
Edaravone	6.3 mg/kg	6.80 ± 0.66^#^
Deferoxamine	70 mg/kg	4.60 ± 1.17

Data are expressed as the mean ± SEM, *n* = 5. ^*∗∗*^*P* < 0.01 vs. sham group. ^#^*P* < 0.05 vs. model group.

**Table 3:** Effect of RAP on Fn, FHC, and FLC protein expression in rats with CIRI induced by MCAO.

Group	Fn	FHC	FLC
Sham	52.238 ± 4.77	0.481 ± 0.07	0.620 ± 0.04
Model	79.32 ± 4.94^*∗∗*^	0.933 ± 0.04^*∗∗*^	0.938 ± 0.04^*∗∗*^
RAP granule (2.5 g/kg/d)	44.766 ± 6.42^##^	0.575 ± 0.07^##^	0.475 ± 0.09^##^
RAP injection (2 ml/kg/d)	52.086 ± 4.86^##^	0.465 ± 0.11^##^	0.668 ± 0.09^#^
Calycosin (10 mg/kg/d)	55.802 ± 3.18^#^	0.703 ± 0.08^#^	0.607 ± 0.08^##^
Edaravone (6.3 mg/kg/d)	69.564 ± 7.00	0.562 ± 0.08^##^	0.612 ± 0.07^##^
Deferoxamine (70 mg/kg/d)	54.046 ± 8.96^##^	0.523 ± 0.06^##^	0.505 ± 0.06^##^

Data are expressed as the mean ± SEM, *n* = 5. ^*∗∗*^*P* < 0.01 vs. sham group. ^#^*P* < 0.05 and ^##^*P* < 0.01 vs. model group.

**Table 4:** Effect of RAP on LTCC protein expression in rats with CIRI induced by MCAO.

Group	Dose (g·kg^−1^)	LTCC
Sham		86.134 ± 3.77
Model		105.292 ± 1.45^*∗∗*^
RAP granule	2.5 g/kg	90.89 ± 6.31^#^
RAP injection	2 ml/kg	90.22 ± 5.66^#^
Calycosin	10 mg/kg	99.458 ± 0.88
Edaravone	6.3 mg/kg	94.432 ± 4.23
Deferoxamine	70 mg/kg	94.824 ± 1.87

Data are expressed as the mean ± SEM, *n* = 5. ^*∗∗*^*P* < 0.01 vs. sham group. ^#^*P* < 0.05 vs. model group.

**Table 5:** Effects on Tf, TfR, DMT1, TRPC6, and FPN1 in rats with CIRI induced by MCAO.

Group	Tf	TfR	DMT1	TRPC6	FPN1
Sham	34.032 ± 2.21	62.834 ± 4.59	78.772 ± 9.21	47.284 ± 6.32	95.252 ± 3.03
Model	81.342 ± 7.09^*∗∗*^	98.41 ± 1.10^*∗∗*^	103.354 ± 0.97^*∗∗*^	94.036 ± 2.62^*∗∗*^	63.832 ± 6.10^*∗∗*^
RAP granule	50.776 ± 3.08^##^	49.764 ± 10.15^##^	86.286 ± 5.36^#^	56.57 ± 10.53^##^	81.296 ± 3.35^#^
RAP injection	62.93 ± 6.69^#^	63.328 ± 2.69^##^	71.254 ± 6.45^##^	67.334 ± 10.31^#^	80.212 ± 5.90
Calycosin	70.198 ± 8.62	66.638 ± 6.94^##^	88.046 ± 6.28	62.706 ± 8.00^#^	74.014 ± 5.21
Edaravone	55.828 ± 6.41^##^	66.584 ± 4.64^##^	96.762 ± 1.14	69.536 ± 13.00	83.408 ± 7.97^#^
Deferoxamine	74.832 ± 4.65	74.164 ± 9.22^#^	89.366 ± 3.83	66.376 ± 7.69^#^	80.142 ± 6.42

Results of the IHC data are expressed as the mean ± SEM, *n* = 5. ^*∗∗*^*P* < 0.01 vs. sham group. ^#^*P* < 0.05 and ^##^*P* < 0.01 vs. model group.

## Data Availability

The data used in this study are available from the corresponding author on reasonable request.
